The article "Synthesis and Anticancer Activity of Di(3-thienyl)methanol and Di(3-thienyl)methane" was published in 2012. Journal: Molecules.

# Synthesis and Anticancer Activity of Di(3-thienyl)methanol and Di(3-thienyl)methane 

**DOI:** 10.3390/molecules171011456

**Published:** 2012-09-27

**Authors:** Nagendra Kumar Kaushik, Hong Seon Kim, Young June Chae, Young Nam Lee, Gi-Chung Kwon, Eun Ha Choi, In Tae Kim

**Affiliations:** 1 Plasma Bioscience Research Center, Kwangwoon University, Seoul 139-701, Korea; 2 Department of Chemistry, Kwangwoon University, Seoul 139-701, Korea

**Keywords:** thienyl derivatives, T98G gliomas, HEK cells

## Abstract

Di(3-thienyl)methanol (**2**) and di(3-thienyl)methane (**3**) have been synthesized and screened against the T98G (brain cancer) cell line. Treatment induced cell death (MTT and macro-colony assay), growth inhibition, cytogenetic damage (micronuclei formation), were studied as cellular response parameters. Treatment with the compounds enhanced growth inhibition and cell death in a concentration dependent manner in both T98G and HEK (normal) cell lines. At higher concentrations (>20 µg/mL) the cytotoxic effects of the compounds were highly significant. The effect on clonogenic capacity and micronuclei formation observed after treatment of cells. Amongst the compounds, compound **2** exhibited potent activity against T98G brain cancer cells. Despite potent *in vitro* activity, both compounds exhibited less cytotoxicity against normal human HEK cells at all effective concentrations.

## 1. Introduction

The development of new cancer therapeutic agents is one of the fundamental goals in medicinal chemistry. One newer strategy for the research on new antimicrobial therapeutic agents has been the use of N- and S-containing small heterocyclic compounds. In the race to synthesize new antiproliferative drugs, thiophene derivatives have attracted a great deal of attention amongst the scientific community due to their therapeutic uses. The thienyl nucleus is also the core structure of a great number of cancer growth inhibitors. Thiophene and the thienyl core have attracted the attention of the scientific community due to their therapeutic uses as antimicrobial [1], anti HIV [2], PTP1β inhibitors [3], tyrosine kinase inhibitor [4], antioxidant [5,6], anti-inflammatory [5,6], analgesic [5], anti-nociceptive [6], antitubercular [7], antiarrhythemic [8], anticonvulsant [8], antiparasitic [9], anticancer agents [10,11,12] and metabolic stability in cells [13]. The present work is in continuation of our search for small medicinal active molecules and evaluation of their biological activity. In this present study we describe anticancer activity of two dithienyl derivatives: di(3-thienyl)methanol (**2**) and di(3-thienyl)methane (**3**) against T98G brain cancer cells. The cytotoxicity of the synthesized compounds on normal cells were assessed using the HEK cell line, which resembles developing neuron and neuronal stem cells and is also mentioned as good model for neuroscience studies [14]. Based on this background, we have used HEK normal cells as a model for brain normal cells in this study.

## 2. Results and Discussion

### 2.1. Synthesis

We have synthesized di(3-thienyl)methanol (**2**) and di(3-thienyl)methane (**3**) and studied their anticancer effects (Scheme 1 and Figure 1). The structures of compound **2** and **3** are clearly supported by their ^1^H, ^13^C-NMR spectra and microanalysis.

**Scheme 1:** Synthesis of compound **2** and **3**.

**Figure 1:** Energy minimized 3D structure of di(3-thienyl)methanol (**2**) and di(3-thienyl)methane (**3**). Red, yellow, white color ball represents oxygen, sulfur and hydrogen atoms respectively. Pink balls represent lone pairs on the oxygen atom.

### 2.2. MTT Assay

The 3-(4,5-dimethylthiazol-2-yl)-2,5-diphenyltetrazolium bromide (MTT) cell proliferation assay has been widely accepted as a reliable way to measure the cell proliferation rate and cell death [15,16]. The data obtained by MTT assay show that compounds **2** and **3** have inhibitory effects on the growth of T98G and HEK cells in dosage-dependent manners. Compounds **2** and **3** can inhibit 50% T98G cell growth (IC_50_) obviously in the 60–200 µg/mL range after 24, 48 and 72 h of the treatment (Figure 2). Maximum inhibitory effect was shown by compound **2** on T98G cells after 72 h of treatment, however compound **3** also effectively inhibits the growth of T98G cells at all the concentrations (0.7–2,500 µg/mL) and without any time dependent effects (Figure 2). Overall compound **2** was the most potent one, having significant a inhibitory effect on T98G cells growth. Both compounds are less toxic to the HEK cells with 75%–97% viability at 60 µg/mL concentration at all time intervals, which further increased by decreasing the concentration of the compounds (Figure 2). For further studies, we have selected compound **2** on the basis of its significant toxicity against T98G brain cancer cells.

**Figure 2:** % Viability evaluated from MTT assay on T98G brain cancer and normal HEK cells treated with thienyl derivative for 24, 48, and 72 h.

### 2.3. Growth Kinetics Assay

Figure 3 shows the growth kinetics of T98G cells treated with compound **2**. Cell proliferation kinetics have been studied at 24, 48, 72 h after compound treatment, following trypsinization and counting total cells per plate by using a trypan blue dye and hemocytometer. Data obtained from the growth kinetics assay shows that compound **2** has inhibitory effects on the growth of T98G cells in a concentration dependent manner. 

**Figure 3:** Growth kinetics of T98G cells at 24, 48 and 72 h after treatment by compound **2** at 2.2–200 µg/mL concentrations. Untreated cells are taken as control and all values given as mean (±SE) of three independent experiments, n = 3.

It was also noted that the cells exposed to 2.2 and 6.6 µg/mL concentrations show less growth inhibitory effects than those treated with 20, 60 and 200 µg/mL concentration. Maximum effect was shown by 200 µg/mL concentration of compound **2**, which inhibits the growth of cells up to 93% at 48 and 72 h after treatment and its viability range was 7%–8%. In the case of 20 and 60 µg/mL exposures, we found 45%–60% cells death at all time intervals. Cell morphology analysis revealed that shape and size of viable cells were also affected by treatment of compound **2** (Figure 4). From Figure 4 it is found that there was remarkable differences in shape and size of treated cells at 2.2, 20, 60 and 200 µg/mL after treatment.

**Figure 4:** Morphology of compound **2** treated T98G brain cancer cells at 24 h after treatment. Cells were treated at concentration 2.2, 6.6, 20, 60 and 200 µg/mL.

### 2.4. Clonogenic Assay

The clonogenic assay shows the effect of compound **2** on the colony-forming capacity and survival of exponentially growing T98G cells. We have used the clonogenic assay for confirming the growth inhibition results of compound **2**. Clonogenic assay or colony formation assay is an *in vitro* assay based on the ability of a single cell to grow into a colony. Only a fraction of seeded cells retains the capacity to produce colonies after cytotoxic drug treatment. As observed in Figure 5, the surviving fraction of T98G cells has been drastically decreased after its treatment by compound **2**. Compound **2** treatment enhances cell death and also inhibits colony formation capability in the T98G cell population in a concentration dependent manner. After treatments with different concentrations (2.2–200 µg/mL), the surviving fraction of T98g cells declines, as evidenced by the reduction in the number of colonies formed. Even at low doses, 2.2, 6.6 and 20 µg/mL exposure of compound **2** shows a significant decline in colony survival and the surviving fractions was found to be 0.85, 0.71 and 0.58, respectively. However, a significant drastic decline in their surviving fraction could be observed after exposure to 60 and 200 µg/mL treatment and their surviving fractions were found to be 0.32 and 0 (zero), respectively. This shows that these treatments significantly inhibit the colony formation capabilities of brain cancer cells at all the dosages. 

**Figure 5:** Effect of compound **2** on colony forming capacity and survival of exponentially growing T98G cell lines studied by macro colony assay. Data presented are mean values from three independent observations, n = 3.

### 2.5. Micronucleus Assay

In recent years, the *in vitro* micronucleus (MN) assay has become an attractive tool for measuring genotoxicity by physical and chemical agents, due to its capacity to detect clastogenic and aneugenic events, simplicity of scoring, accuracy, multipotentiality and wide applicability in different cell types. For measuring micronucleus, we have treated T98G cells with compound **2** under similar conditions and concentrations to those which were used in earlier experiments on growth kinetics and the clonogenic assay. After treatment by compound **2**, cell cultures were grown for a 24 and 48 h in order to allow chromosomal damage leading to the formation of micronuclei in bi- or multinucleated interphase cells. 

Figure 6 shows the micronucleus frequency at 24 and 48 h for T98G brain cancer cell after treatment with 2.2–60 µg/mL concentration of compound **2**. The frequency of untreated cells with micronuclei were in the range of 3.5%–3.9%; whereas the treatment with 2.2 µg/mL does not induce any significant level of micronuclei formation in T98G cells, and the range of micronucleus is 3.8–3.9. However, micronuclei frequency increased from 3.5% (control) to 5.6%, 6.21% and 7.7% for 6.6, 20 and 60 µg/mL concentration treated cells, respectively, at 24 h of culture. However, it was increased further at 48 h of culture as 6.6, 20 and 60 µg/mL concentrations of compound **2** further increased micronuclei frequency from 3.9% (control) to 5.9%, 6.43% and 7.9%, respectively. Micronuclei shown in compound **2** treated T98G cells were formed by DNA strand breaks generated during the faulty excision repair process. The remaining unsealed DNA leads to the formation of micronuclei in subsequent mitosis, and cells with micronuclei are found to be associated with loss of reproductive capacity.

**Figure 6:** Comparison between micronucleus (MN) frequencies at 24 and 48 h in human T98G cells treated with compound **2**. Whereas ‘Control’ is micronuclei frequency of untreated cells.Results are measured *in vitro* both in mononucleated cells and binucleated cells in cultures. These cells shown with one or many micronucleus were scored for MN frequency. The data represents mean ± SEM, n = 3.

### 2.6. *In Silico* Pharmacokinetics

For a molecule to be a probable drug, besides having a good biological activity, it must have nice pharmacokinetic accessibility in biological systems. To access the pharmacokinetic profile of the synthesized molecule, we used the well validated *in silico* tools: Osiris, Chemaxon and Catalyst. These tools have been validated with almost 7,000 drug molecules available in market. The analysis of theoretical toxicity risks for the thienyl derivatives using the OSIRIS program shows that all compounds were less toxic and can be used as a therapeutic molecules (Figure 7). As these compounds are considered for oral delivery, they were submitted to the analysis of Lipinski ‘rule of five’, druglikness and drug score by using the Catalyst software (Table 1).

**Figure 7:** *In silico* drug safety analysis for thienyl derivatives by Osiris software.

Our results pointed that all effective compounds fulfill this rule and their druglikness property such as molecular weight (180–196), Log P (2.38–3.13), nHBA (0–1), nHBD (0–1) and number of rotatable bonds (rotb) (2) were better than commercial drugs (Table 1). Finally, we evaluated thienyl derivative **2** as a potential drug by calculating druglikeness and drug-score. Druglikeness, which is related to the similarity with trade drugs (−1.28–1.29). Drug score of all derivatives was in the range of 0.46–0.56. Among the both thienyl compounds, **2** showed the best values of drug-score (0.56) with a lower toxicity effect, which suggests it should be considered for further *in vivo* exploration.

**Table 1:** Pharmacokinetic parameters (Catalyst, Chemaxon and Osiris softwares).

Compounds	nHba	nHbd	nrotb	MW	cLog P	Druglikeness	Drug Score
2	1	1	2	196	2.38	−1.29	0.56
3	0	0	2	180	3.13	−2.28	0.47

## 3. Experimental

### 3.1. General

The MTT (3-[4,5-dimethylthiazol-2-yl]-2,5-diphenyltetrazolium bromide), bisbenzimidazole derivative Hoechst-33342 (bis-benzimide(2-[4-ethoxyphenyl]-5-[4- methyl-1-piperazinylpiperazinyl]-2,5-bi-1H-benzimidazole)trihydrochloride), Hank’s balanced salt solution (HBSS), Dulbecco’s modified phosphate buffered saline (PBS), Dulbecco’s modified eagle’s medium (DMEM), fetal calf serum (FCS), N-[2-hydroxyethyl]piperazine-N-[2-ethanesulfonic acid] (HEPES) buffer, propidium iodide (PI), Ribonuclease-A (RNase-A), trihydro-chloride, propidium iodide and trypsin were obtained from the Sigma Chemical Co., USA. All other chemicals used in the present study were of analytical grade. 

### 3.2. Preparation of Di(3-thienyl)methanol (2)

3-Bromothiophene (**1**, 60 g, 0.36 mol) was added into a solution of *n*-butyllithium (0.36 mol) in THF (120 mL) at −78 °C and a solution of the ethyl formate (13.63 g, 0.184 mol) in THF (60 mL) was added dropwise while maintaining the temperature between −78 and −70 °C [17]. The mixture was then allowed to warm slowly (over ~1 h) to RT. The resulting mixture was hydrolyzed with 10% aqHCl (76.8 g) with cooling below 0 °C. The organic layer was separated, and the aqueous layer was extracted with CHCl_3_ (300 mL × 3). The combined solutions were dried with Na_2_SO_4_ and concentrated in vacuo. The residue was chromatographed on a short silica gel column (hexane-EA 6:1) to yield a pale-yellow viscous oil, which solidified upon standing. Yield: 88% (31.78 g); m.p. 61–62 °C. ^1^H-NMR (400 MHz, CDCl_3_): 7.19 (dd, 2H, *J* = 5.0, 3.0 Hz), 7.07 (m, 2H), 6.93 (dd, 2H, *J* = 5.0, 1.3 Hz), 5.76 (s, 1H), 3.10 (br s, 1H); ^13^C-NMR (100 MHz, CDCl_3_): 144.71 (2C), 126.26 (2C), 125.94 (2C), 121.50(2C), 68.67. Anal Calcd for C_9_H_8_OS_2_:C, 55.07; H, 4.11 Found: C, 54.88; H,4.17.

### 3.3. Preparation of Di(3-thienyl)methane *(**3**)*

To a well stirred solution of chlorotrimethylsilane (55.34 g, 0.5094 mol) in anhydrous CH_3_CN (240 mL) was added NaI (76.35 g, 0.5094 mol) in one portion. The resulting slurry was stirred for 20 min at 0 °C, and then a solution of corresponding di(3-thienyl) methanol (**2**, 20 g, 0.1018 mol) in CH_3_CN (150 mL) was added dropwise over 30 min to maintain the reaction temperature below 10 °C [18]. The reaction mixture was quenched with aqueous NaOH (10.99 g in 150 mL) extracted with CH_2_Cl_2_ (300 mL × 3), washed with a saturated solution of Na_2_S_2_O_3_·5H_2_O (150 mL), and dried over Na_2_SO_4_. Organic solvents were removed *in vacuo*, and the brown residue was purified by column chromatography (hexane) to yield the pure di(3-thienyl)methane (**3**) as a white solid or pale yellow oil which solidified upon standing. Yield: 90% (16.51 g); m.p. 35–36 °C. ^1^H-NMR (400 MHz, CDCl_3_): 7.38 (dd, 2H), 7.09 (m, 2H), 4.14 (s, 2H); ^13^C-NMR (100 MHz, CDCl_3_): 140.75 (2C), 128.21 (2C), 125.42 (2C), 121.00(2C), 30.89. Anal Calcd for C_9_H_8_OS_2_: C, 59.96; H, 4.47 Found: C, 59.74; H, 4.19.

### 3.4. Human Cell Culture

T98G (brain cancer) and HEK Normal (Human Embryonic Kidney) cells were used in the present studies were purchased from SNU (Seoul, Korea). We were culture these cell line in 75 cm^2^ culture flasks (Corning, New York, NY, USA) using Dulbecco’s modified Eagle’s medium (DMEM) supplemented with 10% fetal bovine serum, 1% nonessential amino acids, 1% glutamine, penicillin (100 IU/mL) and streptomycin (100 mg/mL) (all from Euroclone, UK) or by distributor instructions. All cultures were maintained at 37 °C, 95% relative humidity and 5% CO_2_. Prior to each cytotoxicity test, the cells were harvested using trypsin–ethylenediaminetetraacetic acid (EDTA)–PBS solution (with 0.25% trypsin–0.05mM according to the distributor’s instructions) and diluted at a density of 5 × 10^5^ cells/mL in MTT assays. Stock cultures were passaged every third day after harvesting the cells with 0.05% trypsin and seeding 8 × 10^3^ cells/cm^2^ in tissue culture flasks to maintain the cells in the exponential phase. All experiments were carried out in exponentially growing cells. The cell suspension was seeded into 24-well plates (Corning, New York, NY, USA) at 100 µL well, and incubated for approximately 20–24 h before tests in order to reach confluency. Before the cells were seeded into 24-well plates, the plates were treated with 0.01% poly-D-lysine solution (Sigma-Aldrich, Germany).

### 3.5. *In Vitro* Cell Viability Assay

Cells were seeded in 24-well plates at a concentration of 2–4 × 10^3^ cells/well in 200 μL of complete media and incubated for 24 h at 37 °C in 5% CO_2_ atmosphere to allow for cell adhesion. All assays were performed in two independent sets of quadruplicate tests. Control group containing without treatment was run in each assay. Following after 24, 48 and 72 h of exposure of cells to compound, each well will be carefully rinsed with 200 μL PBS buffer. Cytotoxicity were assessed using MTT (3-[4,5-dimethylthiazol-2yl]-2,5-diphenyltetrazolium bromide). MTT solutions 20 μL (5 mg·mL^−1^dd H_2_O) along with 200 μL of fresh, complete media were added to each well and plates were incubated for 3 h [19]. Following incubation, the medium were removed and the purple formazan precipitate in each well were sterilized in 200 μL DMSO. Absorbances were measured using microplate reader at 570 nm and results were expressed as % viability which is directly proportional to metabolic active cell number. Percentage (%) viability was calculated as:


% Viability = OD in sample well/OD in control well × 100

### 3.6. Cell Growth Kinetics Assay

Cells were seeded at 7,000–10,000 cells/cm^2^ in 90–120 mm Petri dishes or flasks, and their proliferation kinetics will be studied at 24, 48, 72 h after treatment by compounds, following trypsinization and counting total cells per flask/disc by using a Neubauer hemocytometer.

### 3.7. Clonogenic Survival Assay

Clonogenic assay or colony formation assay is an *in vitro* cell survival assay based on the ability of a single cell to grow into a colony. The colony is defined to consist of at least 50 cells. The assay essentially tests every cell in the population for its ability to undergo “unlimited” division [20]. Clonogenic assay is the method of choice to determine cell reproductive death after treatment with ionizing radiation, but we can also be used to determine the effectiveness of drug molecules. Only a fraction of seeded cells retains the capacity to produce colonies before or after treatment, cells will be seeded out in appropriate dilutions to form colonies in 1–3 weeks. After harvesting with 0.05% trypsin, 150–400 (depending on the treatment) cells will be plated 10–14 h before treatment in DMEM at 37 °C. Cultured cells will be treated with doses 20 to 100 ug/ml of compounds. After the treatment, cells will be incubated in dark under humidified, 5% CO_2_ atmosphere at 37 °C for 8–10 days to allow colony formation. Colonies will be fixed with methanol and will be stained with 1% crystal violet. Colonies of more than 50 cells will be counted and the surviving fraction (SF) will calculated. Clonogenic survival curves will be constructed from three independent experiments by least-squares regression fitting averaged survival levels. 

### 3.8. Micronuclei Formation

The purpose of the micronucleus assay is to detect those chemical and physical agents which modify chromosome structure and segregation in cells [21]. For measuring micronucleus we treated T98G cells by compound under similar conditions as we used in earlier experiments for growth kinetics and clonogenic assay. After treatment by compound, cell cultures are grown for a 24 and 48 h to allow chromosomal damage to lead to the formation of micronuclei in bi- or multinucleated interphase cells. Air-dried slides containing acetic acid–methanol (1:3 V/V) fixed treated cells were stained with Hoechst-33342 (10 µg/mL in PBS (0.1M), disodium phosphate (0.45 M) buffer containing 0.05% Tween-20 detergent). Slides were examined under the fluorescence microscope using an UV excitation filter. Fluorescent nuclei were visualized using a blue emission filter. Cells containing micronuclei were counted from >1,000 cells by employing the criteria of Countrymen and Heddle [21]. 

The fraction of cells containing micronuclei, called the M-fraction (%) or MN frequency was calculated as follows:


M-fraction (%) = *N*m/*N*t × 100

where Nm is the number of cells with micronuclei and *N*t is the total number of cells analyzed. Since, micronuclei formation is linked to cell proliferation, the micronuclei frequencies were normalized with respect to the cell numbers.

### 3.9. *In Silico* Pharmacokinetic Screening

To evaluate pharmacokinetic profile descriptors such as cLogP (octanol/water partition coefficient) and LogS (water solubility) were calculated using the Osiris Property Explorer on-line system [22]. The thienyl derivatives were submitted to *in silico* absorption, distribution, metabolism, excretion, and toxicity (ADMET) screening, using the Osiris program. Values of druglikeness are based on the occurrence frequency of each fragment of the molecule in commercial drugs while the drug-score evaluates the compound’s potential to qualify for a drug and is related to topological descriptors, fingerprints of molecular druglikeness, structural keys and other properties such as cLog P and molecular mass [22,23]. *In silico* theoretical safety analysis is also evaluated by Osiris software, whereby a score of 1 means a drug is safe and a score < 1 means a drug molecule is theoretically toxic in use. The pharmacokinetic profile, important for a good oral bioavailability of a compound, was also evaluated according to the Lipinski’s ‘rule-of-five’ by using the Catalyst and Chemaxon softwares, which analyse features that a drug should present to allow the absorption and permeation across the membranes and states molecular weight < 500 Daltons (Da), calculated octanol/water partition coefficient (cLogP) < 5, number of hydrogen-bond acceptors (nHba) < 10, and number of hydrogen-bond donors(nHbd) < 5 [22,23], as well as a fifth rule added later, which infers the number of rotatable bonds < 10.

## 4. Conclusions

The obtained results for human T98G brain cancer cells were compared with Human Embryonic Kidney (HEK) cells. The compounds were more efficacious on T98G cancer cells and are less toxic to normal human HEK cells. These thienyl derivatives may be regarded as lead structures for a new class of anticancer agents with both drug delivery capability because of small size and capable of chemosensitization. Finally we can conclude that compound **2** and **3** could have the broad dosage ranges of activity against human T98G brain cancer cells. Compound **2** shows significant toxicity on T98G cells and the least toxicity on normal HEK cells. Compound **2** also inhibits the clonogenic capacity of T98G brain cancer cells in a concentration dependent manner. Compound **2** presents the overall best parameters including: (a) high activity against a brain cancer cell line, (b) low cytotoxicity risks in HEK cells, (c) low toxic effect risks in *in silico* analysis, (d) good oral bioavailability according to the Lipinski ‘rule of five’, and (e) better druglikeness and drug-score values, nearly similar or better than some commercial drugs. Studies on the mechanism by which the compound **2** induce antiproliferative effect on T98G brain cancer cells and a wider range of other cancer cell lines are ongoing.
